The article "Folic Acid Protects Melanocytes from Oxidative Stress via Activation of Nrf2 and Inhibition of HMGB1" was published in 2021. Journal: Oxid Med Cell Longev.

# Folic Acid Protects Melanocytes from Oxidative Stress via Activation of Nrf2 and Inhibition of HMGB1

**DOI:** 10.1155/2021/1608586

**Published:** 2021-12-07

**Authors:** Pengran Du, Shaolong Zhang, Shuli Li, Yuqi Yang, Pan Kang, Jiaxi Chen, Tianwen Gao, Chunying Li, Qian Zhang, Weigang Zhang

**Affiliations:** Department of Dermatology, Xijing Hospital, Fourth Military Medical University, No. 127 of West Changle Road, Xi'an, Shaanxi 710032, China

## Abstract

Vitiligo is a cutaneous depigmentation disease due to loss of epidermal melanocytes. Accumulating evidence has indicated that oxidative stress plays a vital role in vitiligo via directly destructing melanocytes and triggering inflammatory response that ultimately undermines melanocytes. Folic acid (FA), an oxidized form of folate with high bioavailability, exhibits potent antioxidant properties and shows therapeutic potential in multiple oxidative stress-related diseases. However, whether FA safeguards melanocytes from oxidative damages remains unknown. In this study, we first found that FA relieved melanocytes from H_2_O_2_-induced abnormal growth and apoptosis. Furthermore, FA enhanced the activity of antioxidative enzymes and remarkably reduced intracellular ROS levels in melanocytes. Subsequently, FA effectively activated nuclear factor E2-related factor 2 (Nrf2) pathway, and Nrf2 knockdown blocked the protective effects of FA on H_2_O_2_-treated melanocytes. Additionally, FA inhibited the production of proinflammatory HMGB1 in melanocytes under oxidative stress. Taken together, our findings support the protective effects of FA on human melanocytes against oxidative injury via the activation of Nrf2 and the inhibition of HMGB1, thus indicating FA as a potential therapeutic agent for the treatment of vitiligo.

## 1. Introduction

Vitiligo is an acquired depigmentation dermatosis with an estimated prevalence of 1% worldwide [1]. To date, the reason for the loss of epidermal melanocytes as the key event in vitiligo is still unclear, which hinders the development of effective therapeutic strategies [2]. Nevertheless, recent studies have indicated the involvement of oxidative stress in the pathogenesis of vitiligo [3]. Along with the deficiency of antioxidant system of melanocytes, especially nuclear factor E2-related factor 2 (Nrf2) pathway that is a master regulator of antioxidative response [4, 5], reactive oxygen species (ROS) such as hydrogen peroxide (H_2_O_2_) is excessively accumulated in vitiligo [6]. Accordingly, melanocytes are susceptible to ROS-induced apoptosis in vitiligo [3, 5]. Moreover, ROS facilitates the release of high-mobility group protein B1 (HMGB1) that belongs to damage-associated molecular patterns (DAMPs) with strong proinflammatory effects from melanocytes [7–10]. HMGB1 subsequently causes the production of chemokines in adjacent keratinocytes and the maturation of dendritic cells (DCs) in a paracrine way, which ultimately promotes the formation of cytotoxic T cells (CTLs) that undermine melanocytes in vitiligo [7]. Therefore, oxidative stress plays a vital role in vitiligo via not only direct oxidative damages on melanocytes but also triggering cutaneous T cell response that targets melanocytes.

The article "Folic Acid Protects Melanocytes from Oxidative Stress via Activation of Nrf2 and Inhibition of HMGB1" was published in 2021. Journal: Oxid Med Cell Longev.

Folic acid (FA), a synthetic oxidized form of folate with high bioavailability, is well known for its protective effect against neural tube defects [11]. FA digested at intestine is ultimately converted to 5-methyltetrahydrofolate with the help of methylenetetrahydrofolate reductase (MTHFR) and then involved in the remethylation of homocysteine (Hcy) to methionine [12]. In 2014, our group reported an association between single-nucleotide polymorphisms (SNPs) in *MTHFR* gene and vitiligo susceptibility [13]. Furthermore, Hcy was observed to accumulate in vitiligo and induce the apoptosis of melanocytes via endoplasmic reticulum stress [14]. These findings indicate that the disruption of folate metabolism plays a role in the pathogenesis of vitiligo. Notably, some recent studies have found that FA possesses excellent antioxidant property and is effective in maintaining cellular redox status [15, 16]. However, the effect of FA on melanocytes under oxidative stress in vitiligo has not been investigated before.

Herein, we initially observed that FA did protect melanocytes from oxidative damages. Furthermore, the influence of FA on the antioxidant response of melanocytes was evaluated. In addition, the effect of FA on the status of HMGB1 in melanocytes under oxidative stress was also investigated in the present study.

## 2. Materials and Methods

### 2.1. Cell Culture and Treatment

The immortalized normal human epidermal melanocyte cell line PIG1 (a gift from Dr. Caroline Le Poole, Loyola University, Chicago, USA) was maintained in Medium 254 (M254500, Gibco, USA), supplemented with human melanocyte growth supplement (Gibco) and 5% fetal bovine serum at 37°C amid 5% CO_2_. Oxidative stress was induced by adding H_2_O_2_ (7722841, Sigma-Aldrich, USA) at 800 or 500 *μ*M into the culture medium for 48 h. To determine the protective effect of FA (F8758, Sigma-Aldrich, USA) on melanocytes against oxidative damages, FA and H_2_O_2_ were added simultaneously into the culture medium of PIG1 cells at indicated concentrations.

### 2.2. CCK8 Assay

Cell viability was evaluated by using a CCK8 kit (C008, 7Sea biotech, China) according to manufacturer's manual. Generally, PIG1 cells were seeded into 96-well plates at the density of 2 × 10^4^ cells per well before further treatments as indicated. Next, 10 *μ*l of CCK8 solution was added to each well, and the cells were further incubated at 37°C for 2 h. The optical density (OD) was measured at 450 nm by Model 680 Microplate Reader (BioRad, USA). All experiments were performed in triplicate.

The article "Folic Acid Protects Melanocytes from Oxidative Stress via Activation of Nrf2 and Inhibition of HMGB1" was published in 2021. Journal: Oxid Med Cell Longev.

### 2.3. Apoptosis Assay

Cell apoptosis was measured using Annexin V-FITC/PI kit (A005, 7 Seabiotech, China). Briefly, the treated PIG1 cells were stained according to manufacturer's instructions and then detected by flow cytometry (Beckman Coulter, USA) and analyzed with Expo32 software (BeckmanCoulter, USA).

### 2.4. Western Blot Assay

Whole cell lysates were extracted with RIPA Buffer (P0013C, Beyotime, China). Nuclear/cytoplasmic fractionation was separated using the Nuclear and Cytoplasmic Protein Extraction Kit (P0028, Beyotime, China) according to manufacturer's instructions. Protein concentration was measured using the BCA Protein Assay kit (23225, Thermoscientific, USA). Equal amounts of protein were separated by SDS-PAGE (Bio-Rad, USA) and transferred to polyvinylidene difluoride membranes (Millipore, USA). Membranes were blocked in 5% nonfat milk for 2 h and incubated overnight at 4°C in primary antibodies diluted with PBS containing 1% BSA, including mouse anti-human *β*-actin (8H10D10) (1 : 5000, 3700, Cell Signaling Technology, USA), rabbit anti-human LaminA/C (1 : 1000, 10298–1-AP, Proteintech, China), rabbit anti-human Tubulin (1 : 2000, 11224-1-AP, Proteintech, China), rabbit anti-human Bcl-2 (D55G8) (1 : 1000, 4223, Cell Signaling Technology, USA), rabbit anti-human Bax (D2E11) (1 : 1000, 5023, Cell Signaling Technology, USA), rabbit anti-human cleaved Caspase-3 (Asp175) (5A1E) (1 : 1000, 9664, Cell Signaling Technology, USA), rabbit anti-human Caspase3 (1 : 1000, Lot. 9662, Cell Signaling Technology), rabbit anti-human Nrf2 (1 : 500, ab62352, Abcam, USA), rabbit anti-human Nrf2 (phospho S40) (1 : 5000, ab76026, Abcam, USA), mouse anti-human HO-1 (1 : 500, ab13248, Abcam, USA), rabbit anti-human SOD2 (1 : 2000, ab13533, Abcam, USA), and rabbit anti-human HMGB1 (1 : 500, ab18256, Abcam, USA). After washing, the membranes were incubated at room temperature for 2 h in corresponding peroxidase-conjugated secondary antibodies diluted with PBS containing 1% BSA, including goat anti-rabbit IgG antibody (1 : 5000, AP132P, Sigma-Aldrich, United States) and goat anti-mouse IgG antibody (1 : 5000, AP124P, Sigma-Aldrich, United States). At last, the bands were detected by an enhanced chemiluminescence reagent (Millipore, USA) under Western blotting detection system (Bio-Rad, USA).

The article "Folic Acid Protects Melanocytes from Oxidative Stress via Activation of Nrf2 and Inhibition of HMGB1" was published in 2021. Journal: Oxid Med Cell Longev.

### 2.5. SOD Activity Assay

After cells were lysed, the total protein was extracted to detect the activity of SOD by using Total Superoxide Dismutase Assay Kit with WST-8 (S0101M, Beyotime, China) following manufacturer's instructions.

### 2.6. Measurement of Intracellular ROS

The intracellular ROS was measured using a fluorogenic probe for ROS (CM-H2DCFDA) (C6827, Invitrogen, USA) following the protocol reported previously [17]. Briefly, PIG1 cells were seeded into 6-well plates with a density of 5 × 10^5^ cells. After indicated treatments, 10 *μ*M of DCFH-DA was added for 30 min, and then, cells were collected for detection of fluorescence intensity of DCF via flow cytometry (Beckman Coulter, USA).

### 2.7. Immunofluorescence Assay

PIG1 cells were grown in single-layer glass slides (801002, NEST Biotechnology, China) at a density of 5000 cells per dish. After indicated treatments, cells were washed by PBS and fixed with 4% paraformaldehyde. Cells were permeabilized for 15 min in PBS supplemented with 0.1% Triton X-100 at room temperature and labeled with the primary antibody anti-Nrf2 (1 : 200, ab62352, Abcam, USA) at 4°C overnight and corresponding secondary antibody Cy3-tagged goat anti-rabbit IgG (1 : 1000, ab6939, Abcam, USA) for 1 h at room temperature. At last, cells were incubated with the nuclear dye 40, 6-diamidino-2-phenylindole (DAPI) (1 : 1000, 62247, Thermo Fisher Scientific, USA) for 10 min at room temperature in the dark. The fluorescence was detected by using FV-1000/ES laser confocal microscopy (Olympus, Japan).

### 2.8. Enzyme-Linked Immunosorbent Assay (ELISA)

ELISA was performed using the Human HMGB1 ELISA Kit (Shino-Test, Japan) according to manufacturer's instructions. The absorbance (A450) was measured with a plate reader (Bio-Rad).

### 2.9. Quantitative Real-Time Polymerase Chain Reaction (qRT-PCR)

Total RNA was extracted using Trizol Reagent (15596018, Invitrogen, United States) and then reversely transcribed to cDNA by a PrimeScript RT reagent kit (AK4301, TaKaRa, Japan). The qRT-PCR assay was performed using SYBR PremixEx Taq II (AKA1008, TaKaRa, Japan) with the real-time PCR Detection System (Bio-Rad, United States). The relative mRNA expression was normalized to the *β*-actin gene. The primers used in this study were as follows: HMGB1, forward: AGCCCTCTTCATGTTCCGAAGTGT, reverse: TCATGTCAACACCTGCAGTCCCTT; *β*-actin, forward: TCATGAAGTGTGACGTGGACATC, reverse: CAGGAGGAGCAATGATCTTGATCT.

### 2.10. RNA Interference

PIG1 cells were seeded at 2 × 10^5^ cells per well for 24 h before transfection. Cells were transfected with Nrf2 shRNA or irrelevant shRNA control (GenePharma, China) with Lipofectamine 3000 (Invitrogen) following manufacturer's protocol. The sequences of the shRNAs used in the present study were as follows: shRNA-Nrf2: 5′-GGTTGCCCACATTCCCAAATC-3′; shRNA-Control: 5′-TTCTCCGAACGTGTCACGT-3′.

The article "Folic Acid Protects Melanocytes from Oxidative Stress via Activation of Nrf2 and Inhibition of HMGB1" was published in 2021. Journal: Oxid Med Cell Longev.

### 2.11. Statistical Analysis

Data analysis was performed using GraphPad Prism version 6.0 software (GraphPad Software, San Diego, CA). The two-tailed Student's *t*-test or one-way analysis of variance (ANOVA) was used in our analyses. *P* values less than 0.05 were considered significant. Data represent as mean ± SD for at least three independent experiments.

## 3. Results

### 3.1. FA Protects Melanocytes from Oxidative Stress

CCK8 assay was initially performed to evaluate suitable doses of FA for use in subsequent experiments. As a result, FA at the concentrations of 10 to 500 *μ*M had no significant influence on the growth of PIG1 cells over an incubation course of three days, but high doses (1000 and 3000 *μ*M) of FA showed toxicity on the third day (Figure 1(a)). To investigate the protective effect of FA on melanocytes under oxidative stress, PIG1 cells were treated with FA at a concentration gradient of 25, 50, and 100 *μ*M, respectively, and costimulated with 800 *μ*M H_2_O_2_ for 24 h. It turned out that H_2_O_2_-induced morphologic changes of shortened or disappeared dendrites in PIG1 cells were significantly rescued by the pretreatment with FA at relatively higher doses of 50 or 100 *μ*M (Figure 1(b)). Consistently, FA reversed the inhibited viability of PIG1 cells caused by H_2_O_2_ in a dose-dependent manner (Figure 1(c)).

We went on to investigate whether FA protects melanocytes from apoptosis under oxidative stress. Flow cytometry analysis showed that the proportion of apoptotic PIG1 cells was markedly increased after the treatment with H_2_O_2_, whereas the cotreatment with FA at the concentrations of 50 or 100 *μ*M significantly rescued PIG1 cells from H_2_O_2_-induced apoptosis (Figures 2(a) and 2(b)). Moreover, the upregulated protein levels of proapoptotic Bax and cleaved Caspase-3 and the downregulated protein level of Bcl-2 caused by H_2_O_2_ were all reversed by cotreated FA (100 *μ*M) in PIG1 cells (Figure 2(c)). Altogether, these results support that FA protects melanocytes from oxidative damages.

### 3.2. FA Potentiates Antioxidant Response in Melanocytes under Oxidative Stress

Next, the influence of FA on the antioxidant system of melanocytes was evaluated. The accumulation of ROS in PIG1 cells treated with H_2_O_2_ was attenuated by the cotreatment with FA at the concentrations of 50 *μ*M or 100 *μ*M (Figures 3(a) and 3(b)). Meanwhile, the repressed activity of superoxide dismutase (SOD), a key antioxidant enzyme that scavenges ROS [17, 18], was significantly reversed by FA at 100 *μ*M in PIG1 cells treated with H_2_O_2_ (Figure 3(c)).

The article "Folic Acid Protects Melanocytes from Oxidative Stress via Activation of Nrf2 and Inhibition of HMGB1" was published in 2021. Journal: Oxid Med Cell Longev.

Since Nrf2 plays a central role in the antioxidant system of melanocytes [3, 5], we then evaluated the effect of FA on the activation of Nrf2 pathway. As shown by our Western blot analysis, the cotreatment of FA promotes the expressions of Nrf2, phosphorylated Nrf2 (p-Nrf2) that acts as a transcriptional factor as well as SOD2 and heme oxygenase-1 (HO-1) that are antioxidant proteins transcriptionally regulated by p-Nrf2 in PIG1 cells treated with H_2_O_2_ (Figure 3(d)). Subsequent detection of nuclear and cytosolic Nrf2 separately disclosed that FA induced the translocation of Nrf2 from cytoplasm to nucleus in H_2_O_2_-treated PIG1 cells (Figure 3(e)), which was further supported by immunofluorescence assay (Figure 3(f)). Collectively, our findings indicate that FA enhances antioxidant response in melanocytes under oxidative stress.

### 3.3. FA Prevents Melanocytes from Oxidative Damages via Activating Nrf2 Pathway

To decide whether the protective effect of FA on melanocytes under oxidative stress is dependent on the activation of Nrf2, Nrf2 was silenced by transfecting PIG1 cells with short hairpin RNA (shRNA) of Nrf2 (interference efficiency shown in Figure 4(a)). It was found that FA failed to eliminate intracellular ROS in H_2_O_2_-treated PIG1 cells as long as Nrf2 was deficient (Figures 4(b) and 4(c)). Moreover, Nrf2 knockdown abolished the protection of FA against H_2_O_2_-induced apoptosis on PIG1 cells (Figures 4(d) and 4(e)). Further Western blot assay observed that Nrf2 knockdown abrogated FA-induced upregulation of HO-1 and SOD2 in H_2_O_2_-treated PIG1 cells (Figure 4(f)). Altogether, these findings demonstrate that the activation of Nrf2 pathway mediates the protection of FA on melanocytes against oxidative damages.

### 3.4. FA Reduces the Release of HMGB1 from Melanocytes under Oxidative Stress

Given the proinflammatory role of HMGB1 secreted by melanocytes under oxidative stress in the immune pathogenesis of vitiligo as described before, the effect of FA on the status of HMGB1 in ROS-triggered melanocytes was examined at last. Consistent with our previous report [7], H_2_O_2_ prominently increased the mRNA and protein levels of HMGB1 in PIG1 cells; both of which, however, were repressed by the addition of FA into the culture (Figures 5(a) and 5(b)). Additionally, the cotreatment with FA successfully prevented the release of HMGB1 from H_2_O_2_-treated PIG1 cells (Figure 5(c)). Therefore, FA is of promising potential in inhibiting oxidative stress-induced inflammatory response mediated by HMGB1 in vitiligo.

The article "Folic Acid Protects Melanocytes from Oxidative Stress via Activation of Nrf2 and Inhibition of HMGB1" was published in 2021. Journal: Oxid Med Cell Longev.

## 4. Discussion

Oxidative stress is convincingly a key pathogenetic factor of vitiligo and contributes to its onset and progression [19]. Excessive ROS production and insufficient antioxidant response jointly lead to the destruction of melanocytes in vitiligo [18], which prompts us to seek for measures that rebalance the redox homeostasis of melanocytes. Previous studies have shown that FA keeps the survival of astrocytes and purkinje neurons by decreasing ROS level [20, 21]. Meanwhile, rats treated with FA could obtain high levels of antioxidative enzymes like SOD and low ROS levels [16], indicating that FA potentiates antioxidant system both *in vitro* and *in vivo*. The current study further showed that FA was able to protect melanocytes from oxidative injury by lowering intracellular ROS levels and upregulating HO-1 and SOD2, both of which were reported deficient in vitiligo melanocytes [3, 5]. Further studies using H_2_O_2_-induced vitiligo animal model [22] are needed to confirm the protective effect of FA on melanocytes from H_2_O_2_-triggered oxidation *in vivo*.

Apoptosis is the main form of cell death for melanocytes under oxidative stress [18]. Bcl-2 family proteins including prosurvival Bcl-2 and proapoptotic BAX are the key regulators of apoptosis pathway, in which Caspase-3 acts as a classical executor protein [23]. Herein, FA exhibited potent antiapoptotic ability in human melanocytes under oxidative stress. We previously found that FA protected melanocytes from Hcy-induced apoptosis [14]. Interestingly, Li et al. and Zhou et al. observed that FA inhibited aging-induced apoptosis in astrocytes and neurocytes, respectively, suggesting that FA could suppress apoptosis in various conditions [15, 24]. Additionally, our study showed the upregulation of Bax, the downregulation of Bcl2, and the inhibition of Caspase-3 activation in melanocytes undergoing oxidative stress following FA treatment, indicating that the antiapoptotic capacity of FA may result from decreasing cleaved Caspase-3 through modulating the ratio of Bax to Bcl-2 expression in oxidative injured melanocytes.

Nrf2 is a vital antioxidant regulator that functions as a potent transcriptional activator [4, 25]. Under physiological conditions, Nrf2 is localized primarily in the cytoplasm and bound by Kelch-like ECH-associated protein 1 (Keap1) that hinders the activation of Nrf2 [26]. In response to oxidative stress, Nrf2 is disengaged from its binding to Keap1 and translocated into the nucleus, where Nrf2 potentiates the transcription of antioxidant response elements (AREs) and induces a battery of antioxidant proteins [27]. Nrf2 pathway plays a crucial role in protecting human melanocytes from oxidative stress as demonstrated by our previous studies [4, 5, 28, 29]. Melanocytes in vitiligo are deficient of the activity of Nrf2 and thus more vulnerable to oxidative stress, and reintroduction of Nrf2 pathway is expectedly accompanied with improved survival of melanocytes under oxidative stress [5]. The activation of Nrf2 pathway is characterized by the phosphorylation of Nrf2, the nuclear translocation of Nrf2, and the expression of antioxidant proteins including SOD2 and HO-1 [30], all of which were observed in FA-treated melanocytes by our study. Further knockdown of Nrf2 abolished the protection of FA on melanocytes against oxidative damages, supporting that the antioxidant effect of FA is dependent on Nrf2 pathway in melanocytes. In parallel with our results, Cao et al. found that FA promoted the translocation of Nrf2 from cytoplasm to nucleus and elevated HO-1 expression in rats with spontaneous hypertension [31]. Consistently, the deficiency of folate in fish gills was accompanied with decreased expression of Nrf2 [32]. All of these findings indicate FA as a strong activator of Nrf2 that can be applied extensively.

The article "Folic Acid Protects Melanocytes from Oxidative Stress via Activation of Nrf2 and Inhibition of HMGB1" was published in 2021. Journal: Oxid Med Cell Longev.

Apart from directly killing melanocytes, oxidative stress is known to ignite inflammatory response that ultimately undermines melanocytes in vitiligo [3]. One of the most important mediators of inflammation in vitiligo is HMGB1 released from melanocytes primed by ROS [7]. As a proinflammatory DAMP molecule, HMGB1 acts on its receptors, including several toll-like receptors and receptor for advanced glycation end products (RAGE), and initiates the second wave of protein kinase cascade activation, which generates a positive feedback mechanism to maintain and amplify inflammatory response [33]. Accordingly, the therapies targeting HMGB1 directly or disrupting its binding to proinflammatory receptors may be effective in alleviating inflammation [34]. Sun et al. found that FA-derived drugs disrupted the binding of HMGB1 to receptors and suppressed HMGB1-induced TNF release in human macrophages [35]. Beyond this previous report, our study showed that FA dramatically reduced the mRNA level, protein level, and secretion level of HMGB1 in H_2_O_2_-treated melanocytes, implicating that FA could inhibit oxidative stress-triggered cutaneous inflammation mediated by HMGB1 in vitiligo. In addition, Dong et al. has demonstrated that oxidative damages mediated by HMGB1 could be alleviated with the activation of Nrf2 that further inhibits the expression of HMGB1 [36]. Therefore, the FA-mediated inhibition of HMGB1 in melanocytes observed in the present study was probably mediated by Nrf2 pathway activated by FA.

The article "Folic Acid Protects Melanocytes from Oxidative Stress via Activation of Nrf2 and Inhibition of HMGB1" was published in 2021. Journal: Oxid Med Cell Longev.

The serum level of folate is generally normal in vitiligo patients [37], but recent clinical investigations have confirmed the deficiency of folate in the patients given the phototherapy of narrow-band ultraviolet B (NB-UVB) [38], which is one of the most effective treatments currently applied to vitiligo [39]. Accordingly, taking supplementary FA has been recommended for vitiligo patients on phototherapy, especially for women of childbearing age [40]. Although the results of previous studies are mixed regards to the effect of FA supplementation in vitiligo patients [41], the present study demonstrates FA as an effective agent that protects melanocytes from oxidative damages via its antioxidant and anti-inflammatory capability. Further clinical studies with larger sample size are thus encouraged to evaluate the therapeutic potential of FA for vitiligo.

## Figures and Tables

**Figure 1:** FA attenuated H_2_O_2_-induced oxidative damages in PIG1 cells. (a) The growth of PIG1 cells treated with different concentrations of FA over three days was determined by CCK8 assay. (b, c) PIG cells were treated with different concentrations of FA and 800 *μ*M H_2_O_2_ simultaneously for 48 h. The morphological features of melanocytes were detected by microscope (b). Each field shown is a representative image of at least nine similar fields from three independent experiments. Scale bar = 200 *μ*m. Cell viability was determined by CCK8 assay (c). All data are presented as the mean ± SD across three independent experiments. ^∗^*P* < 0.05, ^∗∗^*P* < 0.01; ns: not significant.

**Figure 2:** FA protected PIG1 cells from H_2_O_2_-induced apoptosis. PIG1 cells were exposed to 800 *μ*M H_2_O_2_ and FA at indicated concentrations for 48 h simultaneously. (a, b) The percentage of apoptotic cells was determined by flow cytometry assay. Bar graphs represent the mean values of flow cytometry data. (c) Effects of FA on H_2_O_2_-induced expressions of Bcl-2, Bax, Casepase-3, and cleaved Caspase-3 were determined via Western blot. *β*-Actin was detected as loading control. Bar graphs represent the quantification of Bcl-2/Bax ratio and cleaved/full length Caspase-3 ratio via gray intensity analysis across three replicate experiments. All data are presented as the mean ± SD across three independent experiments. ^∗^*P* < 0.05, ^∗∗∗^*P* < 0.001; ns: not significant.

**Figure 3:** FA potentiated the antioxidant response in H_2_O_2_-treated PIG1 cells. PIG1 cells were exposed to 800 *μ*M H_2_O_2_ and FA at indicated concentrations for 48 h simultaneously. (a, b) Intracellular ROS level was determined by flow cytometry assay. Bar graphs represent the mean values of the fluorescence intensity of ROS level. (c) The activity of antioxidant enzyme SOD was examined via using a specialized kit. (d) Effects of FA on H_2_O_2_-induced expressions of Nrf2, p-Nrf2, SOD2, and HO-1 were determined via Western blot. *β*-Actin was detected as loading control. (e, f) The nuclear/cytoplasmic distribution of Nrf2 was detected via Western blot (e) and immunofluorescence (f), respectively. Lamin A/C and tubulin were detected as loading controls in western blot assay. Nrf2 was stained with Cy3 (red) and nuclei were counterstained with DAPI (blue) in fluorescence assay. Scale bar = 10 *μ*m. All data are presented as the mean ± SD across three independent experiments. ^∗^*P* < 0.05, ^∗∗^*P* < 0.01, ^∗∗∗^*P* < 0.001; ns: not significant.

The article "Folic Acid Protects Melanocytes from Oxidative Stress via Activation of Nrf2 and Inhibition of HMGB1" was published in 2021. Journal: Oxid Med Cell Longev.

**Figure 4:** Nrf2 knockdown abolished the protective effects of FA on PIG1 cells against oxidative damages induced by H_2_O_2_. PIG1 cells were transfected with the shRNA against Nrf2 or control shRNA for 24 h and then treated with H_2_O_2_ and FA at indicated concentrations for 48 h. (a) The interference efficiency of Nrf2 shRNA was evaluated via Western blot. *β*-Actin was detected as loading control. (b, c) Intracellular ROS level was determined by flow cytometry assay. Bar graphs represent the mean values of the fluorescence intensity of ROS level. (d, e) The percentage of apoptotic cells was determined by flow cytometry assay. Bar graphs represent the mean values of flow cytometry data. (f) The expressions of Nrf2, p-Nrf2, SOD2, and HO-1 were determined via Western blot. *β*-Actin was detected as loading control. ^∗^*P* < 0.05, ^∗∗^*P* < 0.01, ^∗∗∗^*P* < 0.001; ns: not significant.

**Figure 5:** FA inhibited the production of HMGB1 in PIG1 cells treated with H_2_O_2_. (a) The mRNA level of HMGB1 normalized to *β*-actin in PIG1 cells treated with H_2_O_2_ and FA at indicated concentrations for 24 h was determined via qRT-PCR. (b) The protein level of HMGB1 in PIG1 cells treated with H_2_O_2_ and FA at indicated concentrations for 48 h was determined via Western blot. *β*-Actin was detected as loading control. (c) The secretion level of HMGB1 from PIG1 cells treated with H_2_O_2_ and FA at indicated concentrations for 72 h was determined via ELISA. All data are presented as the mean ± SD across three independent experiments. ^∗^*P* < 0.05.

## Data Availability

The data used to support the findings of this study are available from the corresponding author upon request.

## Abbreviations

Nrf2: Nuclear factor E2-related factor 2
ROS: Reactive oxygen species
HMGB1: High-mobility group protein B1
DAMP: Damage-associated molecular pattern
DC: Dendritic cell
CTL: Cytotoxic T cell
FA: Folic acid
MTHFR: Methylenetetrahydrofolate reductase
Hcy: Homocysteine
SNP: Single-nucleotide polymorphism
p-Nrf2: Phosphorylated Nrf2
SOD2: Superoxide dismutase 2
HO-1: Heme oxygenase-1
shRNA: Short hairpin RNA
Keap1: Kelch-like ECH-associated protein 1
ARE: Antioxidant response element
RAGE: Receptor for advanced glycation end products
NB-UVB: Narrow-band ultraviolet B
Bax: B cell lymphoma 2-associated X protein
Bcl-2: B cell lymphoma-2
OD: Optical density
H_2_O_2_: Hydrogen peroxide
PI: Propidium iodide
SDS-PAGE: Sodium dodecyl sulfate-poly-acrylamide gel electrophoresis
PBS: Phosphate buffer solution
DAPI, 4′: 6-Diamidino-2-phenylindole
ANOVA: One-way analysis of variance.
